This article has been retracted.

# Diagnostic Value of FTO Combined with CEA or CYFRA21-1 in Nonsmall Cell Lung Cancer

**DOI:** 10.1155/2021/1436088

**Published:** 2021-10-14

**Authors:** Liqun Shang, Wei Zhang, Hua Wu, Runmiao Wu, Ruilin Chen

**Affiliations:** Department of Respiratory and Critical Care Medicine, Shaanxi Provincial People's Hospital, Xian 710068, China

## Abstract

**Objective:**

To explore the diagnostic value of FTO combined with CEA or CYFRA21-1 for nonsmall cell lung cancer (NSCLC) and to provide a theoretical basis for molecular diagnosis of NSCLC.

**Methods:**

Totally, 60 patients with nonsmall cell lung cancer (NSCLC) treated in our hospital between Feb. 2018 and Feb. 2019 were enrolled into the patient group (Pat group) and 50 healthy individuals with normal physical examination results in our hospital over the same time span into the control group (Con group). Serum of each participant was collected, and then qRT-PCR was adopted for quantification of serum FTO and the chemiluminescence method for quantification of serum CEA and CYFRA21-1. Additionally, corresponding ROC curves were drawn for diagnostic value analyses of FTO, CEA, and CYFRA21-1 in NSCLC and Cox regression analysis was performed for analysis of independent factors impacting the patients' 3-year prognosis.

**Results:**

The Pat group presented notably higher FTO, CEA, and CYFRA21-1 levels than the Con group (all *P* < 0.05), and patients with a high FTO level faced notably higher probabilities of stage III + IV and lymph node metastasis (LNM) (both *P* < 0.05). Additionally, according to ROC curve-based analysis, with a high level in patients with NSCLC, FTO had high specificity and sensitivity in diagnosing NSCLC; joint detection of it with CEA or **C**YFRA21-1 demonstrated a higher sensitivity in NSCLC diagnosis and presented a higher specificity in diagnosing early NSCLC compared with detection of CEA or **C**YFRA21-1 alone. According to Cox regression analysis, clinical stage, LNM, and FTO were independent risk factors impacting the prognosis of patients with LC (all *P* < 0.05).

**Conclusion:**

FTO presents a high level in NSCLC cases, and joint detection of it with CEA or CYFRA21-1 delivered a higher specificity in diagnosing NSCLC in contrast to detection of CEA or **C**YFRA21-1 alone, so the joint detection is worth popularizing in clinical scenarios.

## 1. Introduction

Lung cancer (LC) has always been intractable as a leading cause of death from cancer worldwide [1]. With a gradually growing incidence worldwide, it has ranked first among all kinds of male tumours in terms of incidence, and its incidence among females has also been greatly rising [2]. LC can fall into small cell lung cancer (SCLC) and nonsmall cell lung cancer (NSCLC) in light of its classification, of which NSCLC is the most frequently seen type of clinical LC, taking up to over 85% [3]. At the current stage, the pathogenesis of NSCLC is still under exploration. According to one investigation, smoking history, asbestos exposure, and malnutrition will all raise the incidence of NSCLC [4]. Despite various treatments against NSCLC, such as surgery, chemotherapy, and radiotherapy [5], patients with it still suffer an unfavorable 5-year overall survival (OS) rate due to its late diagnosis and drug resistance to cytotoxicity and the absence of feasible and reliable biomarkers for its diagnosis as well as prognosis [6]. Accordingly, the identification of novel diagnostic biomarkers or therapeutic targets is paramount to the control of tumours.

Epigenetics has become a primary research field over the past several years [7]. According to prior research [8], DNA and histone modification are the focuses in epigenetics. A growing number of studies have revealed various modifications of mRNAs during 5-capping and 3-tailing 4–6 under exon splicing [9], such as N6-methyladenosine (m6A) and N1-methyladenosine (m1A), as well as pseudouridine methylation [10]. These modifications can splice, nucleate, stabilize, and translate mRNAs and further impact their metabolic process, thus changing gene expression. Up to now, 171 RNA modifications have been discovered [11]. M6A, as one crucial modifier, is the most abundant among various eukaryotic mRNAs and lncRNAs 8–10 [12, 13]. FTO is a pivotal demethylase as a nucleoprotein of the superfamily of AlkB-associated nonheme iron and 2-oxoglutaric acid-dependent oxygenase [14]. Ding et al. [15] have discovered that FTO activates cell migration via mRNA demethylation and thus accelerates the progression of lung adenocarcinoma (LA) cells. However, few studies have been conducted on FTO in LC. CEA is a carcinoembryonic antigen, a broad-spectrum tumour marker, but because of its low specificity and sensitivity, it can only reflect the existence and progression of malignant tumors to a certain extent.

Accordingly, this study verified the clinical value of FTO combined with CEA in NSCLC with collected clinical samples to offer potential auxiliary diagnostic indexes to LC diagnosis in clinical scenarios.

## 2. Methods and Materials

### 2.1. Clinical Data

Totally, 60 NSCLC patients (35 males and 25 females, a mean age of (61.1 ± 5.9) years) treated in our hospital between Feb. 2018 and Feb. 2019 were enrolled into the patient group (Pat group), and 50 healthy individuals ((28 males and 22 females, a mean age of (60.2 ± 6.7) years) with normal physical examination results in our hospital over the same time span were enrolled into the control group (Con group). No notable disparity was found between the two groups in age and gender (both *P* > 0.05). The inclusion criteria of patients: (1) patients who were diagnosed as LA via pathological examination/imaging examination and met the staging criteria for NSCLC of the 8th edition of Union for International Cancer Control (UICC) [16]; (2) patients who were newly diagnosed and untreated; (3) patients who did not receive surgical resection, radiotherapy, chemotherapy, molecular targeted therapy, and immunotherapy before enrollment; (4) those who provided signatures on informed consent forms after being apprised of the study. The exclusion criteria of patients: (1) patients with other tumours and patients reluctant to cooperate with follow-up; (2) those with estimated survival time <1 month. This study was in conformity with the Declaration of Helsinki [17].

### 2.2. Specimen Processing

After 30 min still standing, peripheral blood specimens from each patient were subjected to 10 min centrifugation (8 cm, 3000/rpm) for obtaining serum for subsequence analyses, and the remaining samples were conserved at −80°C.

### 2.3. qRT-PCR Assay

Total RNA acquired by TRIzol reagent (Invitrogen company, USA) with sterile and RNase-free surroundings under guidelines was identified to understand its degradation, and the RNA concentration and purity were quantified via NanoDrop (Thermo Scientific). The design and synthesis of FTO primers were conducted by Shanghai Sangon Biotech Co., Ltd. The total RNA was subjected to reverse transcription via a TransScript® Two-Step RT-PCR SuperMix Kit (TransGen Biotech, Beijing, CN) for collecting cDNA that was then treated by PCR amplification under the system configured in the light of the kit guidelines. The amplification was conducted in a system containing cDNA (1 *μ*L), TransTaq® HIFI PCR SuperMix II (12.5 *μ*L), upstream primer (0.5 *μ*L), and nuclease-free water (25 *μ*L), as well as downstream primer (0.5 *μ*L), under predenaturation (94°C, 3 min), followed by 40 cycles of denaturation (94°C, 30 s) and annealing (60°C, 30 s), as well as extension (72°C, 30 s). FTO primer sequence: F: TTTAAGGTGCCAGTCACGA, R: AGTATGGCCGACATTCTGG. FTO was quantified via 2^−△△CT^ (internal reference: GAPDH) [18].

### 2.4. Quantification of CEA and CYFRA21-1

The chemiluminescence method was adopted for quantifying serum CEA and CYFRA21-1 with one automatic biochemical analyzer (ABC AU5800).

### 2.5. Follow-Up of Patients

A follow-up was performed to the patients at the 1^st^, 3^rd^, 6^th^, 9^th^, and 12^th^ months in the first year after discharge, and patients who were enrolled early should be reviewed every 4 months for outpatient electronic medical records and telephone numbers in the second to third years.

### 2.6. Outcome Measures

Primary outcome measures: serum FTO and CEA, as well as CYFRA21, were compared between the Pat group and the Con group, and the value of the three in NSCLC diagnosis was analyzed.

#### 2.6.1. Secondary Outcome Measures

The patients were assigned to corresponding high and low expression groups in the light of median FTO and CEA, as well as CYFRA21-1, and associations of the three with clinical data of LC patients were evaluated. In addition, Cox regression analysis was conducted to clinical data of patients for analysis of independent factors impacting the patients' 3-year prognosis. Kaplan–Meier (K-M) survival curves were drawn for independent factors.

### 2.7. Statistical Analyses

This study utilized SPSS21.0 for statistical analyses of the abovementioned index data and GraphPad Prism 8.0 for visualizing them into corresponding figures. The study expressed measurement data by mean ± SD and conducted their intergroup comparison via the independent-samples T test, and also expressed counting data by *n* (%), and conducted their intergroup comparison via the *χ*2 test. Receiver operating characteristic (ROC) curves were drawn for diagnostic value analyses of FTO, CEA, and CYFRA21-1 in NSCLC, and the K-M method was adopted for analysis of patients' survival. *P* < 0.05 denotes a notable difference.

## 3. Results

### 3.1. FTO, CEA, and CYFRA21-1 in NSCLC Cases

This study quantified serum FTO and CEA, as well as CYFRA21-1, in NSCLC patients and found their higher expression in the patients than that in the Con group (*P* < 0.05; Figure 1).

### 3.2. Associations of FTO and CEA, As Well As CYFRA21-1, with Clinical Data of NSCLC Patients

We analyzed the associations of FTO and CEA, as well as CYFRA21-1, with clinical data of NSCLC patients and assigned them into corresponding high and low expression groups in the light of the median expression of the three. According to analysis, patients with a high FTO level faced notably higher probabilities of stage III + IV and lymph node metastasis (LNM), and CEA was notably bound up with the clinical stage and tumour type of patients with a high CYFRA21-1 level (all *P* < 0.05; Tables 1–3).

### 3.3. Value of FTO and CEA, As Well As CYFRA21-1, in NSCLC Diagnosis

For determining the value of FTO and CEA, as well as CYFRA21-1, in diagnosing NSCLC, we drew corresponding ROC curves and found they were all highly favorable diagnostic indexes of clinical NSCLC because their areas under the curves (AUCs) were all larger than 0.8 in diagnosing NSCLC (Figures 2(a)–2(c)). In addition, joint detection of FTO with CEA or CYFRA21-1 delivered a higher sensitivity in diagnosing NSCLC in contrast to detection of CEA or **C**YFRA21-1 alone (Figures 2(d)–2(e)).

### 3.4. Value of FTO and CEA, As Well As CYFRA21-1, in Diagnosing Early NSCLC

According to analysis of clinical stage, we discovered a certain value of FTO, CEA, and CYFRA21-1 in clinical staging of NSCLC. We classified the NSCLC patients into early-stage patients (stage I, *n* = 17) and middle- and late-stage patients (stage II-IV, *n* = 43) in the light of their clinical stages and analyzed the value of FTO and CEA, as well as CYFRA21-1, in diagnosing early NSCLC by drawing ROC curves. According to the results, in diagnosing early NSCLC, FTO had an AUC of 0.817, while CEA and CYFRA21-1 had AUCs of 0.678 and 0.716, respectively, in it (Figures 3(a)–3(c)). In addition, joint detection of FTO with CEA or CYFRA21-1 delivered a higher specificity in diagnosing early NSCLC in contrast to detection of CEA or **C**YFRA21-1 alone (Figures 3(d)–3(e)).

### 3.5. Value of FTO and CEA, As Well As CYFRA21-1, in Diagnosing NSCLC with LNM

We also found patients with a high FTO level faced a higher probability of NSCLC with LNM. For confirming the value of FTO in diagnosing NSCLC with LNM, we drew corresponding ROC curves and found that in diagnosing NSCLC with LNM, FTO had an AUC of 0.718, while CEA and CYFRA21-1 had AUCs of 0.600 and 0.631, respectively (Figures 4(a)–4(c)).

### 3.6. Cox Regression Analysis

We collected clinical indexes of patients and conducted Cox regression analysis to them for analyzing influencing factors of LC patients' 3-year prognosis. According to Cox regression analysis, clinical stage, LNM, and FTO were all independent risk factors impacting LC patients' prognosis (all *P* < 0.05; Table 4). We also visualized the correlations of FTO, clinical stage, and LNM with patients' 3-year survival into figures (all *P* < 0.05; Figures 5(a)–5(c)).

## 4. Discussion

NSCLC is a malignant tumour with the highest mortality and morbidity worldwide, and its treatment entails strong diagnosis schemes and prognostic indicators [19, 20]. Our study verified an increase of FTO in NSCLC cases via assays and found the unfavorable prognosis of patients with a high FTO level and the ability of FTO to serve as a possible diagnostic index for NSCLC, clinical stage, and lymphatic metastasis.

According to prior research [21], early intervention can prolong the survival of patients. Research has found the significance of biological indicators of patients before therapy for the evaluation of patients' disease severity and efficacy prediction, as well as survival [22]. Therefore, looking for prognostic markers and intervening in advance can prolong the survival of patients. Tumour markers are specific substances synthesized and secreted by cancer cells, which are often adopted as indexes for early diagnosis and prognosis of tumours, with notable elevations in patients with a tumour [22, 23]. CEA is a nonspecific glycoprotein component of cancer cells, with a notably high level in various malignant tumours such as those in the digestive system and respiratory system [24]. CYFRA21-1 can strengthen the decomposition of intercellular connexin and weaken the adhesion between epithelial cells [25]. Recent research has revealed the key functions of CEA and CYFRA21-1 in NSCLC diagnosis and their roles as crucial clinical indexes for the diagnosis [26]. The two have demonstrated a high specificity in NSCLC diagnosis, but their sensitivity in it is unfavorable. Accordingly, raising their sensitivity in NSCLC diagnosis is paramount.

DNA methylation is one crucial mechanism in tumour research [27]. M6A methylation is the most frequently seen form of mRNA modification, which takes a pivotal part in the development of tumours through posttranscriptional regulation [28]. According to one recent study [29], the imbalance in regulatory proteins of m6A methylation can induce the metabolic disorder of downstream RNA, strongly affecting tumour development. FTO, as an m6A eraser, can impact regulating transcription through removing methyl groups from nucleotides [30]. Existing research has revealed strongly correlations of FTO with body mass index [31], obesity risk [32], and type 2 diabetes [33]. One research has also reported the participation of FTO in LC development and its potential to be a diagnostic indicator of LC [34, 35]. In our study, we verified the clinical significance of FTO in NSCLC patients through clinical data. According to the results, with high expression in patients with NSCLC, FTO had a high specificity and sensitivity in diagnosing the disease; joint detection of it with CEA or **C**YFRA21-1 demonstrated a higher sensitivity in diagnosing NSCLC compared with detection of CEA or **C**YFRA21-1 alone. The data suggest the potential of FTO to be a diagnostic biomarker for NSCLC.

We also analyzed the association between FTO and clinical data of NSCLC patients and found patients with a high FTO level faced notably higher probabilities of stage III + IV and LNM. The results denote the possible value of FTO in diagnosing early NSCLC and LNM. Therefore, we assigned the patients into different groups in the light of their clinical stage and LNM. The analysis revealed the clinical significance of FTO in diagnosis of early NSCLC and LNM and a higher accuracy of joint detection of FTO with CEA or CYFRA21-1 in diagnosing early NSCLC compared detection of CEA or CYFRA21-1 alone. Finally, we followed up the patients for 3 years to further probe into the independent factors impacting their prognosis and found FTO, clinical stage, and LNM were independent factors. The results imply a strong association of FTO with the prognosis of NSCLC patients and its potential to be a potential prognostic marker of NSCLC.

Our study has confirmed the diagnostic significance of FTO combined with CEA or CYFRA21-1 in NSCLC through analysis, but it is limited due to the short follow-up time, the single sample, and the absence of diagnostic value analysis of FTO in SCLC. Therefore, we hope to further determine the significance of FTO in LC in the follow-up study with different samples and a longer follow-up time.

To sum up, FTO presents a high level in NSCLC cases, and joint detection of it with CEA or CYFRA21-1 delivered a higher specificity in diagnosing NSCLC compared with detection of CEA or CYFRA21-1 alone, so the joint detection is worth popularizing in clinical scenarios.

## Figures and Tables

**Figure 1:** FTO and CEA, as well as CYFRA21-1, in NSCLC cases. (a) Serum FTO in patients with NSCLC. (b) Serum CEA in patients with NSCLC. (c) Serum CYFRA21-1 in patients with NSCLC. ^*∗∗∗*^*P* < 0.001.

**Figure 2:** Value of FTO and CEA, as well as CYFRA21-1, in NSCLC diagnosis. (a) ROC curve of FTO in NSCLC diagnosis. (b) ROC curve of CEA in NSCLC diagnosis. (c) ROC curve of CYFRA21-1 in NSCLC diagnosis. (d) ROC curve of FTO combined with CEA in NSCLC diagnosis. (e) ROC curve of FTO combined with CYFRA21-1 in NSCLC diagnosis. Note: AUC, area under curve.

**Figure 3:** Value of FTO and CEA, as well as CYFRA21-1, in diagnosing early NSCLC. (a) ROC curve of FTO in diagnosing early NSCLC. (b) ROC curve of CEA in diagnosing early NSCLC. (c) ROC curve of CYFRA21-1 in diagnosing early NSCLC. (d) ROC curve of FTO combined with CEA in diagnosing early NSCLC. (e) ROC curve of FTO combined with CYFRA21-1 in diagnosing early NSCLC. Note: AUC, area under curve.

**Figure 4:** Value of FTO and CEA, as well as CYFRA21-1, in diagnosing NSCLC with LNM. (a) ROC curve of FTO in diagnosing NSCLC with LNM. (b) ROC curve of CEA in diagnosing NSCLC with LNM. (c) ROC curve of CYFRA21-1 in diagnosing NSCLC with LNM. Note: AUC, area under curve.

**Figure 5:** Correlations of FTO, clinical stage, and LNM with patients' 3-year survival. (a) Correlation of FTO with 3-year survival based on the K-M survival curve. (b) Correlation of clinical stage with 3-year survival based on the K-M survival curve. (c) Correlation of LNM with 3-year survival based on the K-M survival curve.

**Table 1:** Association of FTO with clinical data of NSCLC patients (*n*, %).

Index	Relative expression of FTO		*P* value
	High expression (*n* = 30)	Low expression (*n* = 30)	
Age			
≥60 years (*n* = 33)	13	20	0.069
<60 years (*n* = 27)	17	10	
Gender			
Male (*n* = 35)	20	15	0.190
Female (*n* = 25)	10	15	
Tumour size			
≥3 cm (*n* = 30)	17	13	0.302
<3 cm (*n* = 30)	13	17	
Clinical stage			
I + II (*n* = 37)	13	24	0.004^*∗*^
III + IV (*n* = 23)	17	6	
Lymph node metastasis			
Yes (*n* = 18)	14	4	0.005^*∗*^
None (*n* = 42)	16	26	
Tumour type			
Squamous cell carcinoma (*n* = 27)	15	12	0.436
Adenocarcinoma (*n* = 33)	15	18	

*Note.* ^*∗*^ *P* < 0.05 denotes a notable difference.

**Table 2:** Association of CEA with clinical data of NSCLC patients (*n*, %).

Index	Relative expression of CEA		*P* value
	High expression (*n* = 30)	Low expression (*n* = 30)	
Age			
≥60 years (*n* = 33)	15	18	0.436
<60 years (*n* = 27)	15	12	
Gender			
Male (*n* = 35)	16	19	0.432
Female (*n* = 25)	14	11	
Tumour size			
≥3 cm (*n* = 30)	18	12	0.121
<3 cm (*n* = 30）	12	18	
Clinical staging			
I + II (*n* = 37)	14	23	0.017^*∗*^
III + IV (*n* = 23)	16	7	
Lymph node metastasis			
Yes (*n* = 18)	10	8	0.573
None (*n* = 42)	20	22	
Tumour type			
Squamous cell carcinoma (*n* = 27)	8	19	0.004^*∗*^
Adenocarcinoma (*n* = 33)	22	11	

*Note.* ^*∗*^ *P* < 0.05 denotes a notable difference.

**Table 3:** Association of CYFRA21-1 with clinical data of NSCLC patients (*n*, %).

Index	Relative expression of CYFRA21-1		*P* value
	High expression (*n* = 30)	Low expression (*n* = 30)	
Age			
≥60 years (*n* = 33)	19	14	0.195
<60 years (*n* = 27)	11	16	
Gender			
Male (*n* = 35)	15	21	0.114
Female (*n* = 24)	15	9	
Tumour size			
≥3 cm (*n* = 30)	12	18	0.121
<3 cm (*n* = 30)	18	12	
Clinical staging			
I + II (*n* = 37)	14	23	0.017^*∗*^
III + IV (*n* = 23)	16	7	
Lymph node metastasis			
Yes (*n* = 18)	12	6	0.091
None (*n* = 42)	18	24	
Tumour type			
Squamous cell carcinoma (*n* = 27)	18	9	0.019^*∗*^
Adenocarcinoma (*n* = 33)	12	21	

*Note.* ^*∗*^ *P* < 0.05 denotes a notable difference.

**Table 4:** Cox regression analysis.

Index	Univariate analysis			Multivariate analysis		
	*P* value	HR value	95% CI	*P* value	HR value	95% CI
Age	0.817	1.081	0.560–2.087			
Gender	0.891	0.955	0.492–1.853			
Tumour size	0.407	0.758	0.394–1.459			
Clinical stage	0.005	2.571	1.330–4.971	0.033	2.073	1.059–4.060
Lymph node metastasis	0.003	0.369	0.189–0.720	0.041	0.487	0.244–0.971
Tumour type	0.133	0.602	0.31–1.167			
FTO	0.001	0.327	0.164–0.651	0.032	0.451	0.217–0.935
CEA	0.551	1.221	0.634–2.349			
CYFRA21-1	0.262	0.687	0.356–1.325			

## Data Availability

The data can be obtained from all the authors upon reasonable request.
